The article "Role of Managerial Ability in Environmental, Social, and Economics Sustainability: An Empirical Evidence from China" was published in 2022. Journal: J Environ Public Health.

# Role of Managerial Ability in Environmental, Social, and Economics Sustainability: An Empirical Evidence from China

**DOI:** 10.1155/2022/8588385

**Published:** 2022-08-23

**Authors:** Muhammad Kaleem Khan, R. M. Ammar Zahid, Khuram Shahzad, Muhammad Jameel Hussain, Mbwana Mohamed Kitendo

**Affiliations:** ^1^Asia-Australia Business College, Liaoning University, Shenyang, China; ^2^School of Accounting, Yunnan Technology and Business University, Kunming, Yunnan, China; ^3^Research Institute of Business Analytics and Supply Chain Management, College of Management, Shenzen University, Shenzen, China; ^4^School of Management, Xian Jiaotong Univesity, Xi'an, China; ^5^Department of Political Science and Public Administration, Dar Es Salaam University, Dar es Salaam, Tanzania

## Abstract

The current study analyzed whether the enhancement in managerial ability accelerates the environmental, social, and economic sustainability practices or not. Using panel data methodology on Chinese listed firms data from 2010 to 2019, we report that CEOs' managerial ability impacts the overall (environmental, social, and economic) sustainability practices of the firms positively. Moreover, we find that social sustainability and economic sustainability also increase with the increase of the CEO's managerial ability in the firm. The results remain robust after several alternative empirical tests. The findings justify the relationship between management skills and sustainability and demonstrate how each one of the sustainability pillars is affected individually. The support for sustainability practices that can be achieved through the communication of management skills is an essential conclusion for practitioners. Findings establish the link between CEO's managerial ability and environmental, social, and economic sustainability performance by taking insights from upper echelon theory.

## 1. Introduction

The consequences of industrialization including depleting supplies, ruined ecosystems, and the misuse of both natural resources and human labor are some of the reasons driving stakeholders to demand greater corporate accountability, especially in terms of sustainability. The United Nations has established 17 global sustainable development goals (SDGs) with 169 related targets, reflecting its commitment to solving global environmental and sustainable development issues. Griggs, et al. [1] highlighted social, environmental, and economic aspects as the main pillars of sustainable development and redefined them to include “development that meets current needs while safeguarding the Earth's life-support system, upon which the welfare of current and future generations is contingent.” Focusing on the firm's “triple bottom line” functioning should be the contemporary approach toward accountability [2]. Sustainability could only be achieved by equally valuing all its aspects (social, environmental, and economic). For this reason, the Global Reporting Initiative's (GRI) sustainability indicators are structured to provide insight into a company's major economic, environmental, and social consequences, as recommended by the GRI's sustainability reporting criteria [3, 4]. Achieving a balance between the sustainability pillars requires a thorough grasp of how society and industrial actions affect the environment, as well as how today's decisions may affect future generations. As a result, a greater understanding and awareness of the concerns surrounding sustainable development is required.

Institutional factors and organizational attributes are found as primary determinants of sustainability by past researchers [5, 6]. However, the trend is shifting now, and some recent research has focused on the chief executive officer (CEO) and its role in transparency and accountability [7]. Under this prism, researchers have tried to link sustainability and CEO traits (e.g., power, educational background, political ideology, gender, age, experience, personality, media exposure, religiosity, leadership style, and experience) [8–10].

This study aims to investigate the relationship between a chief executive officer's (CEO) management ability and the company's sustainability performance (SP). Although a vast body of literature is available separately for sustainability performance and managerial ability, the need is to bridge this relationship. A more extensive examination of the relationship between the CEO's managerial competence and sustainability characteristics is required for a complete understanding. There have only been a few attempts to understand this link. Recently and Yuan et al [5], García‐Sánchez et al [8] have tried to explain the link between CEO's managerial ability and CSR (Corporate Social Responsibility)/Sustainability performance. Still, both of these studies have not digested the sustainability deeper and did not employ a triple-down approach. In contrast, our empirical contribution takes into account three perspectives of sustainability.

Moreover, the above studies did not study the relation between ability and sustainability in developing economies like China, as this study has done. This research discovers numerous aspects of the management ability-sustainability nexus by individually assessing the various components of sustainability. By this, the study presents a multi-faceted view of sustainability on one. It highlights the role of the ability of the corporate level management to make the firm accountable on economic, social, and environmental grounds. This study adds to the body of research concerning the ties between leadership competencies and sustainability dimensions, substantiating statements about the interrelationships and relative importance of various sustainability aspects [11].

We conduct such rigorous research since the existing literature does not cover the influence of the CEO's managerial ability on all three elements of business sustainability. We use the GRI's SP reporting framework to accomplish this. Businesses must disclose both positive and negative results on all aspects of sustainability, assuming that each is equally vital for long-term development, according to sustainability reporting rules (sustainability reporting guidelines, GRI 2006. (Vol. G3)) [2]. This study reveals multiple aspects of the management-sustainability nexus by quantifying the various sustainability features independently [11].

Scientists have examined sustainability from several theoretical vantage points, including resource dependence [12], resource-based [13], stewardship [14, 15], and neo-institutional [16]. But any theory separately falls short in explaining the link completely [2], and no single hypothesis can adequately explain the expected links [17]. Theoretically, our research contributes to different managerial-related, governance-related, and society related different paradigms. Our main hypothesis was developed through upper echelon theory. The upper echelon theory says that a manager's personality is the key determinant of how a company makes decisions. Since it was impossible to ignore the role of different corporate governance systems as mediators in the management-sustainability nexus, agency theory concepts were also used to figure out how managerial competence and sustainability are related. The study also took insights from stakeholder theory [18] in highlighting the multi-faceted view of sustainability. Our findings may also help guide future research: because the projected influence is often focusing on just one aspect of sustainability (either environmental or social), it necessitates assessing the triple bottom line sustainability performance.

Section 2 will discuss the literature review and hypothesis development in detail. Data and Research methodology details are in section 3. Followed by discussions of results and conclusions, respectively in Sections 4 and 5.

## 2. Literature Review and Hypothesis Development

In the literature, several organizational, individual, societal, and institutional elements of SP have been identified. There is a recent drive to explore the influence of CEO conduct on SP [19], based on the idea that CEOs establish the driving mechanism of the organization. In their capacity as chief executive officers, CEOs are responsible for assessing the requirements of all stakeholders and organizing the company's production to satisfy those needs [20, 21]. This is why making sustainability a high priority is essential [22]. Several qualities of CEOs, including their values [23], incentives [24], narcissism [25], career horizon [26], hubris [27], education [28], political ideology [28], have been cited as determinants impacting SP in the literature.

The relationship between CEOMA and SP is well confirmed by the upper echelon theory. This idea says that the strategic decisions and results of businesses are affected by the personalities and skills of the CEOs. [19]. CEOMA is associated with an improved grasp of firm's operation and performance drivers [29, 30], better utilization of organizational resources [31], appraising new business ventures, as well as to deal with uncertainty [5], to comprehend and respond to environmental motivations [27], embracing innovative strategies [32, 33], and take risks [34].

According to Porter [35], managers may prioritize research and development, advertising, and employee training above fulfilling quarterly and yearly goals. When outcomes are unsatisfactory, it is usual practice to alter management [36, 37], and former leaders may have difficulty reentering the workforce [38]. Consistent with the theory that management turnover is proportional to performance [39], firms with more competent management are more likely to implement sustainable practices. Long-term investments in CSR provide delayed and unforeseeable returns [40–42]. CEOs may be less inclined to invest in CSR if doing so may be detrimental to their careers. CEOs with exceptional skills have less need to be concerned about their career fate [29] and are able to ignore pressure to engage in high-returning ventures. Moreover, because of their ability to deal with ambiguity, more successful CEOs are less likely to be intimidated by the uncertainty associated with CSR investment. Since CSR strategy is often long-term and hazy, the capacity of CEOs to affect their firms' CSR actions is vital [5]. Therefore, competent managers are more inclined to undertake CSR activities despite the risks and long-term consequences [43]. According to prior research [5, 30], the CSR investments and performance of a firm are strongly connected with the managerial competence of the CEO.

We suggest that skilled leaders are more likely to prioritize corporate social responsibility. Competent CEOs would choose for more successful CSR initiatives to further enhance sustainability in environmental, social, and economic dimensions [27, 30].

H1: CEO's management skills are positively related to corporate sustainability performance.

### 2.1. Managerial Ability and Social Sustainability

Traditionally, social sustainability has been seen as a government responsibility, but firms are increasingly recognized as significant players. Relationships with employees, consumers, suppliers, and communities are examples of socially sustainable activity. Social sustainability is defined as a system's ability to maintain an adequate level of social well-being. Thus, an organization is socially sustainable when its activities promote future generations' abilities to maintain healthy communities. Some topical topics in social sustainability include child labor, ethical trading, and supply chain management. Although child labor is prohibited in most countries, it is nonetheless widely practiced. Ethical trading means trading with integrity and legality. Among unethical trading, practices are bribery, anti-competitive behavior, corruption, extortionate pricing, unethical marketing, and market power abuse. Many organizations, particularly multinationals, have broad and complex supply lines. Corporate accountability is increasingly demanded, not just for their activities but also for those of their suppliers. Those firms are more likely to avoid social sustainability, which does not employ optimal use of firm resources. The firm's route to long-term competitive advantage is aided by efficient resource usage and market understanding [44]. Firms with CEOs of superior managerial ability make the best utilization of firm resources [31, 45]; thereby, these firms do not need to indulge in antisocial sustainability practices [5].

H2: CEO's management skills are positively associated with social sustainability performance.

### 2.2. Managerial Ability and Environmental Sustainability

Environmental sustainability comprises making responsible decisions and taking action to protect the natural world, with a focus on human life-support [46]. Environmental sustainability has various compelling arguments. Sustainability is crucial from a humanistic standpoint since humans depend on nature for survival and must address the challenges it causes. Climate change, waste, and pollution are among the other environmental issues [47]. A sustainable future is unfairly burdened on future generations, according to the intergenerational argument. Naturalists argue that nature has intrinsic value and should be preserved. While some of these arguments may be more persuasive than others, they all add to a compelling case for environmental sustainability. Given their increased risk aversion, CEOs with weaker managerial competence will make short-term investment decisions, avoiding riskier assets [48]. Short-term investments, low-risk ventures, and quick talent transfer are preferred by less capable CEOs [49]. Keeping all these in mind, we hypothesize that CEOs with superior managerial ability will not hesitate to invest in environmental protection.

H3: CEO's management skills are positively associated with social sustainability performance.

### 2.3. Managerial Ability and Economic Sustainability

The economic dimension of sustainability addresses an organization's impact on local, national, and global economic systems. It implies maximizing existing resources for a business entity so that the organization can function at a given level of activity for many years. The goal is to encourage long-term use of those resources. Economic sustainability involves the long-term viability of the businesses and the stability of the economic system. One of the most critical aspects of economic sustainability is transparency, openness, and authenticity about a corporation's operations and strategy. Transparency allows external stakeholders to assess a corporation's risk exposure. CEOs with superior managerial ability demonstrate deep knowledge of their business, leading to better judgments and estimates; leading to better reporting quality and transparency [31].

H4: CEO's management skills are positively associated with economic sustainability performance.

## 3. Research Methodology

### 3.1. Data Description

Financial and corporate governance data for all 4,132 A-shares issued between 2010 and 2019 on the Shanghai and Shenzhen exchanges were made accessible through a popular Chinese website “ (China Stock Market and Accounting Research).” In 2010, we started collecting data after China's Thousand Talents Plan [50], which assisted in the recruitment of CEOs based on their management skills, was introduced at the end of 2008. Using the HEXUN website, we acquired RKS ratings for every A-share Chinese listed business. The HEXUNRKS rankings are based on the social, environmental, and economic elements, as well as the overall CSR score, of each year's reviewed Chinese enterprises. As far as, we can ascertain, all publicly listed Chinese firms that submit sustainability reports are included. These databases are widely used in Chinese-related research [51, 52]. To limit the risk of outliers, we eliminated financial institutions from the data set and sorted continuous observation variables with a 1% tail. If a company's values were missing for three consecutive years, they were eliminated from consideration. The whole dataset consists of 3,052 enterprises with 20,651 firm-year observations ranging from 1,373 in 2010 to 2,663 in 2018. This dataset is not uniformly distributed across the sampled companies (lowest to highest).

### 3.2. Variables Design

#### 3.2.1. Dependent Variable

Third-party rating agencies such as HEXUNRKS evaluate long-term performance sustainability. Sustainable performance is the total of a company's contributions to CSR programs and their consequences on the environment, society, and bottom line over time. These numbers are continuous variables from the HEXUN database that may take on values between 0 (the lowest rating score) and 100 (the highest rating score) (the highest rating score).

#### 3.2.2. Independent Variable

Management skills are assessed by researchers using a variety of metrics, including corporate size [53], historical stock returns [54], and media evaluation [43, 55]. Measures based on such variables are not thought to be very reliable because they do not have a lot of testing power and most people think they only show talent in management at a median level [45].

This research derives the notion of chief executive officer management skills (CEOMA) from [56]. This statistic is used to assess a CEO's performance compared to others in his or her profession since it assumes that managers who are able to create more with the same set of inputs are more effective. Management ability is intangible and can only be deduced from strategic resource use outcomes. CEOs do two things to improve the appraisal of [45]'s managing skills.. The primary purpose of Data Envelopment Analysis (DEA) was to measure the efficiency of a corporation year-over-year and sector-by-sector. The input and output variables must be specified for this method to function. In order to accomplish this, they accounted for seven distinct figures: (I) cost of goods sold (CGS), (II) selling, general, and administrative expenses (SGA), (III) property, plant, and equipment (PPE), (IV) operating lease (OLease), (V) research and development cost (RD), (VI) goodwill (GW), and (VII) other intangibles (OtherInt). The output variable is the amount of net sales. Initially, they apply DEA to determine the best solution to the following optimization issue:

(1) $$\begin{array}{c} \max_{y}\theta =\frac{\text{Sales}}{\nu_{1}CGS+\nu_{2}SGA+\nu_{3}PPE+\nu_{4}OLease+\nu_{5}R\;D+\nu_{6}GW+\nu_{7}\text{Other Int}}. \end{array}$$

For the efficiency measure, any number between 0 and 1 may be utilized (as determined by the aforementioned DEA model). Due to the dual ownership of the company's efficiency, total production efficiency was split between management and the business as a whole. Six criteria were then identified as either facilitating or inhibiting management help. Company size, market share, positive cash flow, and age (management-supporting parameters), as well as complex multi-segment and international operations, were all regressed against overall company efficiency (factors that hinder management). In particular, they determine the Tobit regression in the following manner:

(2) $$\begin{array}{c} \text{Firm Efficiency}=\beta_{0}+\beta_{1}Ln\left(\text{Total Assets}\right)+\beta_{2}\text{Market Share}+\beta_{3}\text{Positive Free Cash Flow}+\beta_{4}Ln\left(Age\right)+\beta_{5}\text{Business Segment Concenttration}+\beta_{6}\text{Foreign Currency Indicator}+\text{Year Indicators}+\in . \end{array}$$

The Model 2 residual exemplifies managerial expertise. This study employs the decile rank of managerial ability (CEOMA) by year and industry to make the score more comparable across time and industries and to reduce the impact of outliers [45].

### 3.3. Control Variables

To avoid misleading conclusions, we consider a number of firms, board of directors, and chief executive officer-related control criteria. To examine the likelihood that SP is associated with firm performance, growth possibilities, financial health, and firm size, we apply the methodology of [30, 57] and add control variables such as ReturnonAsset, Tobin's *Q*, and Size (log of total assets). The controlled variables Duality (equals 1 if the CEO is also the chairman), CEOGender (equals 1 if the CEO is male), and RetiringCEO (equals 1 if the CEO is 63 or older) are related to the CEO. Board size (the total number of directors on boards), board independence (the proportion of independent directors to total directors), and board meetings (the frequency with which the board meets) are all examples of corporate governance characteristics that may influence management performance (number of board meetings in a year). Following the work of Yuan et al [5], we also employ HHI and FirmAge to analyze the impact of market age on companies (firm age). The Herfindahl–Hirschman Index (HHI) is an indicator of market competition (the sum of the squared market shares of all firms in the same industry, measured at the end of the fiscal year). The financial flexibility of an organization may be controlled by assessing its net operating assets (NOA) and utilizing Altman's z-score (ZScore) to account for the sector and period-level influences, respectively.

### 3.4. Econometric Model

The following model was used to establish the link between CEO's managerial skills and sustainability performance, (SP Social, SP Env, and SP Eco), alternatively.

(3) $$\begin{array}{c} SP_{it}=\beta_{0}+{\text{CEOMA}}_{it}\beta_{\text{CEOMA}}+Z_{it}\beta_{Z}+\in_{it},\\ SP\_{\text{Social}}_{it}=\beta_{0}+{\text{CEOMA}}_{it}\beta_{\text{CEOMA}}+Z_{it}\beta_{Z}+\in_{it},\\ SP\_{\text{Env}}_{it}=\beta_{0}+{\text{CEOMA}}_{it}\beta_{\text{CEOMA}}+Z_{it}\beta_{Z}+\in_{it},\\ SP\_{\text{Eco}}_{it}=\beta_{0}+{\text{CEOMA}}_{it}\beta_{\text{CEOMA}}+Z_{it}\beta_{Z}+\in_{it}. \end{array}$$

*i* and *t* denote the company and the time period, respectively. The vector space of control variables is denoted by *Z*.

### 3.5. Descriptive Statistics

The detailed descriptive statistics are presented in Table 1. The average SP score for Chinese firms came out to be around 23 with minimum score of 0 and maximum of 73. CEO managerial score has a mean of 0.001 with a range from −0.314 to 0.391. Additionally, BoDs in Chinese companies typically consist of 8 to 9 people and have 9 sessions every year. Furthermore, as shown in Table 1, descriptive statistics for the control variables are consistent with prior research [58].

Table 1 provides descriptive statistics for all variables included in the baseline model. Each variable's definition may be found in section 3.2.

## 4. Results and Discussion

### 4.1. Findings on Panel Data Estimations

Panel data estimations using the random effect model technique for models 3–6 present results for the effect of a CEO's managerial ability on sustainability performance as depicted in Table 2. We use a random effect regression model based on the Hausman specification test to examine the impact of *CEOMA* variables on *SP, SP_Social, SP_Env*, and *SP_Eco*. Column 2 in Table 2 shows that the impact of CEO's managerial ability on overall sustainability performance is positive. Specifically, the coefficient is 3.267 at the 1% significance level, implying the positive effect of managerial ability in improving the sustainability-related performance. We hypothesized (H1) that CEO's managerial ability is positively related to sustainability performance. So, our H1 is substantiated. This is in line with our expectations as well as the findings of prior studies like [5, 8, 30, 59]. Previous literature has already identified the importance of superior managerial ability for firms by claiming that managerial ability is a key determinant of firm financial performance [31, 60, 61], we add our findings that managerial ability is also essential for nonfinancial performance (CSR) for the firms. Increasing the management ability increases socially responsible practices and decreases irresponsible behavior related to society, environment, and economy.

We used social SP as the initial dimension for measuring SP. The social performance index is a metric that measures how well a company performs in the areas of labor, human rights, society, and product responsibility. Table 2 shows the findings of the social sustainability analysis (column 3). Our random effect model results reveal that CEOMA is significantly and positively related to SP_Social. The coefficient is 1.401 at a 1% significance level, representing managerial ability has a positive impact on the social dimension of sustainability performance.

The second dimension of sustainability is environmental sustainability (*SP_Env*). This represents the Sustainability performance in relation to environmental practices. The results of *CEOMA* and *SP_Env* are presented in Table 2 (column 4). Our random effect model results reveal that *CEOMA* is negatively but insignificantly related to *SP_Env*. This is contrary to our expectations and hypothesis H3. We hypothesized that increase in managerial ability affects environmental sustainability positively. Despite the fact that these results are contrary to our assumptions, they guide the thinking process toward bettering sustainability strategies. The results are not according to our expectations theoretically, but it is true practically. After the start of thousands of talent programs, Chinese firms performed impressively specifically in terms of growth and market performance; but environmental effects could not be controlled. Still, China is the largest emitter of carbon dioxide and it has the 20 most polluted cities in the world [52, 62, 63]. It means managerial ability is not successful on environmental grounds despite the tremendous efforts of the Chinese government.

The last dimension of sustainability used in this study is economic sustainability. Economic performance is the betterment of the local, national, and international economy. It helps to improve the quality of life of all stakeholders by employing transparency and accountability in entrepreneurial activities. The panel data estimations of economic sustainability are presented in Table 2 (column 4). Our random effect model results reveal that *CEOMA* is significantly and positively related to *SP_Eco* (Coef. 2.907, *p* < 0.01). It implies that an increase in managerial ability increases the economic sustainability practices of Chinese firms.

### 4.2. Robustness Tests

#### 4.2.1. Sensitivity Analysis and Endogeneity Tests

Furthermore, we use various sensitivity analyses to assess the robustness of our primary findings. Our study's sensitivity analysis and endogeneity checks are detailed in Table 3. First, we analyze the impact of CEO managerial skills on future sustainable performance (from Models 3–6) by taking the dependent variables one at a time (*t* + 1) for reverse causality in our regression equations. The results of our random effect panel data analysis corroborate our major findings. We discovered comparable results in our secondary regression analysis as we did in our first regression study. Panel 1 of Table 3 (model 1–4) depicts that CEOMA is significantly and positively associated with overall next year's sustainability performance, social sustainability, and economic sustainability, whereas for environmental sustainability, the coefficient of CEOMA is negative and not significant.

We followed past studies to avoid concerns about endogeneities, simultaneities, and firm-specific heterogeneities in our main regressions [64, 65] and used sGMM (system generalized method of movement) in re‐estimating our results. The results are shown in panel B of Table 4. Our findings are very similar to the primary findings, and they show that our findings are robust to possible spurious correlations caused by heterogeneities or endogeneities. Overall, our sensitivity analysis, endogeneity check, and sample selection test suggest that our primary findings are resistant to the existence of any of these statistical issues.

#### 4.2.2. Alternative Definitions of Managerial Ability

According to existing research, CEOs have a wide range of talents, and business performance is a strong indicator of CEO competence. e.g., [60, 66]. As a robustness test, we re-estimate our models using industry-adjusted return on assets (IndAdjROA) as a surrogate for CEO competency (3–6). For each company year, the IndAdjROA is calculated by subtracting the average industry ROA from the income before unusual items multiplied by the average total assets. The estimated panel data are shown in Table 4. The coefficients of industry-adjusted ROA come out to be significant and positive except for the coefficient of IndAdjROA with *SP_Env* sustainability, which is although positive but not significant. These results confirm our previously obtained results and strengthen our deduction that managerial ability positively impacts sustainability practices along with all its pillars.

## 5. Conclusions and Policy Implementations

This study has linked two important streams; CEO's managerial ability and corporate sustainability performance. The study is critical because it investigates the most important requisite of the organization's leader, “the ability of the CEO.” Moreover, it establishes the stance on how the ability impacts the sustainability practices of the organization. While digging deep, this study presents the triple-down analysis of sustainability performance, i.e., three pillars of sustainability, namely social sustainability, economic sustainability, and environmental sustainability. This is the first study that has (1) researched the relation of a CEO's managerial ability with sustainability in a developing economy and (2) classified sustainability into its main pillars and studied each one with CEO's ability. Using panel data methodology on Chinese listed firms from 2010 to 2019, we report that CEO's managerial ability impacts the overall sustainability practices of the firms positively. Moreover, we find that social sustainability and economic sustainability also increase with the increase of the CEO's managerial ability in the firm. We could not reach any significant relationship between environmental sustainability with managerial ability. Our results remain robust after utilizing various methodologies and definitions. Our findings confirm the upper echelon theory's insights that illustrate that the firm's top leadership characteristics influence firm-level decisions.

There are several policies and regulatory ramifications for our research. There are several policies and regulatory ramifications for our research. One implication of our findings is that Chinese listed firms may need to increase top management's capabilities and expertise (particularly CEOs) to ensure that sustainable policies are effectively implemented. In this instance, the Thousand Talents Plan can be more effective. The Thousand Talents Plan appears to have had a significant impact on the development of modern China since Chinese professionals have joined organizations and made significant contributions to the formulation of strategic policies. The effectiveness of such programs is demonstrated by China's unwavering commitment to environmental and climatic challenges, as evidenced by its signing of the Paris Climate Agreement in 2016. Furthermore, our findings suggest that it is critical to improve CEOs' abilities to foster a positive relationship with and dedication to improving sustainable practices in Chinese businesses. The findings also help strengthen the continuing standard-setting process, especially the in-depth revision of all essential dimensions of sustainability under the new GRI framework.

There are also substantial practical and societal ramifications for policymakers who emphasize CSR. Our research implies that policymakers should consider managers' career concerns when establishing policies to encourage managers to invest in CSR. For example, when assessing the managers' capability, it should be linked with sustainability. It can be achieved by revising the definition of managerial ability. The new definition should be like “managerial ability is a measure to what extent firm utilizes its resources into social, environmental and economic output.” By this, managers will not only utilize their ability and skills on financial performance; relatively sustainable performance will also be equally valued. Our findings are equally applicable to companies that prioritize sustainability. One strategy to encourage sustainable performance is to use incentive systems that compensate CEOs for long-term achievement. One of the most important implications is to educate the firm to perform comprehensive sustainability practices, i.e., social, environmental, and economic sustainability, along with other aspects.

Finally, despite new contributions and significant findings, this study has some limitations that should be acknowledged, and that can also serve as future research areas. First, this study ignored some fundamental aspects of the CEO's traits like his education, financial expertise, and political affiliation with the communist party; all these, among other aspects, influence the managerial ability of China. The best would be to add CEOs' extensive personality index based on the CEO's observable and cognitive characteristics and managerial ability. Second, we have only looked at CEOs from top management. The study can be made more fruitful by including the traits and capabilities of other directors and top management teams. Finally, we only looked at a large sample from a Chinese viewpoint; future studies could provide fresh insights by comparing emerging markets to those in the United States or Europe. The results might differ in other regions as sustainability issues, and managerial capability levels vary from region to region. Our core measure of CEO ability is more dependable and accurate than previous studies' measures; nonetheless, it is probable that our ability measure still captures some features of firms' operational, investing, and financing environments that have not been effectively controlled for. Future research could concentrate on generating more accurate assessments of managerial skills.

## Figures and Tables

**Table 1:** Descriptive statistics.

Variable	Obs	Mean	Std. Dev.	Min	Max
SP	20643	23.331	14.961	0	73.31
CEOMA	20653	0.001	0.157	−314	0.391
BSize	20651	8.569	1.699	0	20
BMeeting	20651	9.611	3.941	0	56
CEOGender	20651	0.938	0.242	0	1
BIndependence	20633	0.374	0.052	0.333	0.571
DebttoAssets	20651	0.415	0.215	0.049	0.944
ROA	20651	0.037	0.065	−299	0.191
RetiringCEO	20651	0.023	0.149	0	1
Duality	20651	0.291	0.454	0	1
HHI	20651	0.319	0.267	0	1
NOA	20651	2.092	2.841	−373	111.143
Size	20651	21.941	1.204	19.639	25.565
TobinsQ	20651	2.038	1.367	0	8.792
AgeofFirm	20651	20.805	5.406	4	41
ZScore	20651	0.838	5.015	−569.231	72.59

**Table 2:** Impact of CEO's Managerial Ability on Social, Environmental, and overall sustainability performance.

	(1)	(2)	(3)	(4)
Variables	*SP*	*SP_Soc*	*SP_Env*	*SP_Eco*
CEOMA	3.627^*∗∗∗*^	1.401^*∗∗∗*^	−0.349	2.907^*∗∗∗*^
	(0.720)	(0.213)	(0.247)	(0.210)
BSize	0.721^*∗∗∗*^	0.0633^*∗∗∗*^	0.263^*∗∗∗*^	0.0471^*∗∗*^
	(0.0792)	(0.0235)	(0.0271)	(0.0231)
BIndependence	11.04^*∗∗∗*^	2.985^*∗∗∗*^	3.458^*∗∗∗*^	−1.060
	(2.281)	(0.660)	(0.783)	(0.658)
BMeeting	−0.105^*∗∗∗*^	−0.00187	−0.0411^*∗∗∗*^	−0.0283^*∗∗∗*^
	(0.0249)	(0.00695)	(0.00857)	(0.00708)
CEOGender	0.435	0.00101	0.245^*∗*^	−0.0218
	(0.425)	(0.123)	(0.146)	(0.123)
RetiringCEO	−1.104^*∗*^	0.0401	−0.371^*∗*^	−0.0999
	(0.616)	(0.172)	(0.212)	(0.175)
Duality	−0.562^*∗∗*^	−0.0953	−0.284^*∗∗∗*^	0.206^*∗∗∗*^
	(0.230)	(0.0662)	(0.0790)	(0.0662)
DebttoAssetsRatio	−2.896^*∗∗∗*^	0.463^*∗∗*^	0.527^*∗∗*^	−4.574^*∗∗∗*^
	(0.633)	(0.185)	(0.217)	(0.183)
ROA	85.44^*∗∗∗*^	14.47^*∗∗∗*^	2.270^*∗∗∗*^	63.33^*∗∗∗*^
	(1.598)	(0.437)	(0.551)	(0.450)
Size	1.891^*∗∗∗*^	0.281^*∗∗∗*^	0.272^*∗∗∗*^	0.731^*∗∗∗*^
	(0.118)	(0.0355)	(0.0405)	(0.0346)
TobinsQ	−0.125^*∗*^	−0.0749^*∗∗∗*^	0.0392	−0.237^*∗∗∗*^
	(0.0716)	(0.0197)	(0.0247)	(0.0202)
AgeofFirm	0.102^*∗∗∗*^	0.0994^*∗∗∗*^	0.0263^*∗∗∗*^	−0.0879^*∗∗∗*^
	(0.0257)	(0.00898)	(0.00872)	(0.00793)
HHI	6.068^*∗∗∗*^	0.446^*∗∗∗*^	2.103^*∗∗∗*^	0.192^*∗∗*^
	(0.314)	(0.0855)	(0.109)	(0.0883)
NOA	−0.136^*∗∗∗*^	−0.0203^*∗∗*^	−0.0285^*∗∗*^	−0.0847^*∗∗∗*^
	(0.0347)	(0.00970)	(0.0119)	(0.00987)
ZScore	−0.0515^*∗∗∗*^	−0.00728	−0.000741	−0.0449^*∗∗∗*^
	(0.0166)	(0.00444)	(0.00573)	(0.00463)
Constant	−33.16^*∗∗∗*^	−6.093^*∗∗∗*^	−9.479^*∗∗∗*^	0.144
	(2.702)	(0.823)	(0.924)	(0.794)
Observations	20,625	20,625	20,625	20,625
Number of id	3,052	3,052	3,052	3,052

Notes: Table 2 presents the random effect panel data estimation results of econometric models 3–6. Definition of each variable can be found in section 3.2. Standard errors are reported in parentheses. ^*∗∗∗*^*p* < 0.01, ^*∗∗*^*p* < 0.05, and ^*∗*^*p* < 0.1.

**Table 3:** Robustness Tests for reverse causality and endogeneity.

	Panel 1				Panel 2			
Variables	(1)	(2)	(3)	(4)	(5)	(6)	(7)	(8)
	SP (*t* + 1)	SP_Soc (*t* + 1)	SP_Env (*t* + 1)	SP_Eco (*t* + 1)	SP	SP_Soc	SP_Env	SP_Eco
l.SP					0.254^*∗∗∗*^			
					(0.00607)			
l.SO_Soc						0.113^*∗∗∗*^		
						(0.00655)		
l.SP_Env							0.303^*∗∗∗*^	
							(0.00631)	
								0.219^*∗∗∗*^
								(0.00437)
CEOMA	3.624^*∗∗∗*^	1.235^*∗∗∗*^	−0.398	2.563^*∗∗∗*^	2.849^*∗∗∗*^	1.559^*∗∗∗*^	−0.102	1.447^*∗∗∗*^
	(0.833)	(0.245)	(0.259)	(0.321)	(0.577)	(0.163)	(0.198)	(0.153)
BSize	0.737^*∗∗∗*^	0.0624^*∗∗*^	0.264^*∗∗∗*^	0.0388	0.469^*∗∗∗*^	0.0219	0.155^*∗∗∗*^	0.0334^*∗∗*^
	(0.0906)	(0.0267)	(0.0282)	(0.0350)	(0.0626)	(0.0176)	(0.0215)	(0.0166)
BInd	10.41^*∗∗∗*^	2.528^*∗∗∗*^	3.353^*∗∗∗*^	−1.208	8.558^*∗∗∗*^	2.169^*∗∗∗*^	2.669^*∗∗∗*^	−1.032^*∗∗*^
	(2.651)	(0.756)	(0.827)	(1.025)	(1.939)	(0.548)	(0.666)	(0.515)
BMeeting	−0.134^*∗∗∗*^	−0.00348	−0.0373^*∗∗∗*^	−0.0681^*∗∗∗*^	−0.0718^*∗∗∗*^	0.0244^*∗∗∗*^	−0.0380^*∗∗∗*^	−0.0126^*∗∗*^
	(0.0298)	(0.00810)	(0.00939)	(0.0116)	(0.0237)	(0.00668)	(0.00813)	(0.00628)
CEOGender	0.191	−0.136	0.286^*∗*^	−0.150	0.282	−0.300^*∗∗∗*^	0.198	0.126
	(0.502)	(0.144)	(0.157)	(0.194)	(0.360)	(0.102)	(0.124)	(0.0957)
RetiringCEO	−1.652^*∗∗*^	−0.362^*∗*^	−0.421^*∗*^	−0.0989	−1.103^*∗*^	−0.0116	−0.264	−0.110
	(0.774)	(0.210)	(0.244)	(0.301)	(0.590)	(0.167)	(0.203)	(0.157)
Duality	−1.049^*∗∗∗*^	−0.104	−0.392^*∗∗∗*^	0.118	−0.399^*∗*^	−0.0842	−0.152^*∗∗*^	0.156^*∗∗∗*^
	(0.274)	(0.0777)	(0.0856)	(0.106)	(0.205)	(0.0579)	(0.0705)	(0.0546)
DebttoAssetsRatio	−3.807^*∗∗∗*^	0.0981	0.792^*∗∗∗*^	−5.980^*∗∗∗*^	−2.455^*∗∗∗*^	0.754^*∗∗∗*^	0.0743	−3.394^*∗∗∗*^
	(0.746)	(0.215)	(0.233)	(0.288)	(0.528)	(0.148)	(0.180)	(0.145)
ReturnonAssets	50.22^*∗∗∗*^	4.866^*∗∗∗*^	3.355^*∗∗∗*^	35.43^*∗∗∗*^	75.69^*∗∗∗*^	15.27^*∗∗∗*^	1.164^*∗∗*^	60.00^*∗∗∗*^
	(2.093)	(0.552)	(0.662)	(0.816)	(1.597)	(0.449)	(0.545)	(0.436)
Size	1.780^*∗∗∗*^	0.158^*∗∗∗*^	0.295^*∗∗∗*^	0.784^*∗∗∗*^	2.008^*∗∗∗*^	0.262^*∗∗∗*^	0.347^*∗∗∗*^	0.748^*∗∗∗*^
	(0.138)	(0.0407)	(0.0427)	(0.0530)	(0.0960)	(0.0262)	(0.0322)	(0.0253)
WobinsQ	0.396^*∗∗∗*^	0.0266	0.108^*∗∗∗*^	0.0189	−0.0657	−0.0486^*∗∗*^	0.0148	−0.127^*∗∗∗*^
	(0.0862)	(0.0228)	(0.0272)	(0.0336)	(0.0711)	(0.0201)	(0.0244)	(0.0189)
AgeofFirm	0.0950^*∗∗∗*^	0.0996^*∗∗∗*^	0.0168^*∗∗*^	−0.0672^*∗∗∗*^	0.0857^*∗∗∗*^	0.0916^*∗∗∗*^	0.0109^*∗∗*^	−0.0402^*∗∗∗*^
	(0.0278)	(0.00961)	(0.00847)	(0.0106)	(0.0155)	(0.00443)	(0.00534)	(0.00415)
HHI	5.995^*∗∗∗*^	0.561^*∗∗∗*^	1.907^*∗∗∗*^	0.485^*∗∗∗*^	4.894^*∗∗∗*^	0.880^*∗∗∗*^	1.368^*∗∗∗*^	0.229^*∗∗∗*^
	(0.389)	(0.101)	(0.123)	(0.152)	(0.331)	(0.0932)	(0.114)	(0.0873)
NOA	−0.182^*∗∗∗*^	−0.0132	−0.0415^*∗∗∗*^	−0.105^*∗∗∗*^	−0.111^*∗∗∗*^	0.0235^*∗∗∗*^	−0.0368^*∗∗∗*^	−0.0608^*∗∗∗*^
	(0.0410)	(0.0112)	(0.0129)	(0.0159)	(0.0308)	(0.00869)	(0.0106)	(0.00818)
ZScore	−0.0226	0.00471	5.61*e* − 05	−0.0245^*∗∗∗*^	−0.0432^*∗∗∗*^	−0.00615	−0.00137	−0.0381^*∗∗∗*^
	(0.0219)	(0.00567)	(0.00697)	(0.00858)	(0.0153)	(0.00432)	(0.00526)	(0.00406)
Constant	−29.85^*∗∗∗*^	−2.899^*∗∗∗*^	−10.13^*∗∗∗*^	−0.191	−38.41^*∗∗∗*^	−5.761^*∗∗∗*^	−9.528^*∗∗∗*^	−5.350^*∗∗∗*^
	(3.090)	(0.931)	(0.958)	(1.190)	(2.126)	(0.588)	(0.726)	(0.553)
Observations	17,071	17,071	17,071	17,071	17,075	17,075	17,075	17,075
Number of id	2,931	2,931	2,931	2,931	2,930	2,930	2,930	2,930
R2	0.37	0.41	0.17	0.57				
AR1 test value					−36.98	−32.98	−31.98	−30.09
AR1 significance					3.83	3.09	3.29	3.28
AR2 test value					−6.34	−6.36	−6.46	−6.63
AR2 significance					2.45	1.98	1.87	1.93

Notes: Panel 1 depicts the random panel data estimation results whereas panel 2 presents system GMM estimation results. Test statistics and standard errors (in parentheses) of all variables in the regressions are asymptotically robust to heteroscedasticity. Definitions of all variables can be found in section 3.2. ^*∗∗∗*^*p* < 0.01, ^*∗∗*^*p* < 0.05, and ^*∗*^*p* < 0.1.

**Table 4:** Robustness Tests: Alternative definition of managerial ability.

	(1)	(2)	(3)	(4)
Variables	*SP*	*SP_Soc*	*SP_En*	*SP_Eco*
IndAdjROA	5.167^*∗∗*^	2.616^*∗∗∗*^	0.0326	2.482^*∗∗∗*^
	(2.041)	(0.526)	(0.723)	(0.513)
BSize	0.864^*∗∗∗*^	0.0583^*∗*^	0.311^*∗∗∗*^	0.0568^*∗*^
	(0.128)	(0.0329)	(0.0454)	(0.0308)
BIndependence	14.15^*∗∗∗*^	3.313^*∗∗∗*^	4.514^*∗∗∗*^	−1.399
	(3.580)	(0.924)	(1.272)	(0.878)
BMeeting	−0.128^*∗∗∗*^	0.00922	−0.0495^*∗∗∗*^	−0.0390^*∗∗∗*^
	(0.0391)	(0.0101)	(0.0139)	(0.00976)
CEOGender	−0.124	−0.140	0.113	−0.0285
	(0.719)	(0.186)	(0.256)	(0.176)
RetiringCEO	−1.160	−0.154	−0.276	−0.317
	(1.112)	(0.287)	(0.394)	(0.278)
Duality	−0.665^*∗*^	−0.0366	−0.322^*∗∗*^	0.187^*∗*^
	(0.402)	(0.104)	(0.143)	(0.0987)
DebttoAssets	−5.947^*∗∗∗*^	0.374	−0.543	−4.706^*∗∗∗*^
	(1.019)	(0.263)	(0.362)	(0.248)
ROA	92.70^*∗∗∗*^	16.02^*∗∗∗*^	4.395^*∗∗∗*^	66.43^*∗∗∗*^
	(2.669)	(0.688)	(0.944)	(0.675)
SizeTA	3.682^*∗∗∗*^	0.355^*∗∗∗*^	0.727^*∗∗∗*^	1.201^*∗∗∗*^
	(0.201)	(0.0519)	(0.0716)	(0.0485)
TobinsQ	−0.331^*∗∗∗*^	−0.0681^*∗∗∗*^	−0.0906^*∗∗∗*^	−0.122^*∗∗∗*^
	(0.0979)	(0.0252)	(0.0346)	(0.0247)
AgeofFirm	0.142^*∗∗∗*^	0.124^*∗∗∗*^	0.0210	−0.0683^*∗∗∗*^
	(0.0485)	(0.0126)	(0.0175)	(0.0110)
HHI	1.868^*∗∗∗*^	0.435^*∗∗∗*^	0.782^*∗∗∗*^	−0.123
	(0.567)	(0.146)	(0.201)	(0.142)
NOA	−0.208^*∗∗∗*^	−0.0369^*∗∗∗*^	−0.0371^*∗∗*^	−0.101^*∗∗∗*^
	(0.0514)	(0.0133)	(0.0182)	(0.0128)
ZScore	−0.0559^*∗∗∗*^	−0.00729	−0.00615	−0.0384^*∗∗∗*^
	(0.0217)	(0.00559)	(0.00766)	(0.00553)
Constant	−69.51^*∗∗∗*^	−7.993^*∗∗∗*^	−17.94^*∗∗∗*^	−10.85^*∗∗∗*^
	(4.655)	(1.202)	(1.660)	(1.114)
Observations	11,007	11,007	11,007	11,007
Number of id	2,147	2,147	2,147	2,147
*R * ^2^	0.389	0.487	0.385	0.329

Notes: Table 4 represent the panel data estimations of the relationship of industry-adjusted ROA with *SO, SP_Soc, SP_Env, and SP_Eco*. Definitions of all variables can be found in section 3.2, except the definition of industry-adjusted ROA, which is given in section 4.2. ^*∗∗∗*^*p* < 0.01, ^*∗∗*^*p* < 0.055, and ^*∗*^*p* < 0.1.

## Data Availability

This study is based on secondary data. All the data are available on the CSMAR data stream.
